# Preventive Effect of Intensive Nursing Intervention of Deep Vein Thrombosis of Lower Extremities in Elderly Patients with Gastrointestinal Tumors after Surgery

**DOI:** 10.1155/2022/2967981

**Published:** 2022-04-26

**Authors:** Yan Li, Fei Xiao

**Affiliations:** ^1^Department of Geriatric Intensive Care Unit Nursing, Sichuan Provincial People's Hospital, University of Electronic Science and Technology of China, Chengdu 610072, China; ^2^Sichuan Translational Medicine Research Hospital, Chinese Academy of Sciences, Chengdu 610072, China

## Abstract

Tumors of the gastrointestinal system, known as gastroenteropapillary neoplasms, are very uncommon yet have a high propensity to progress to cancer. Thromboembolism of the veins (VTE) is a potentially deadly complication of surgery. In the vast majority of cases, deep vein thrombosis (DVT) in the lower extremities is the primary symptom of VTE (DVT). Deep vein thrombosis is more common in critical care units, where the prevalence ranges from 18 to 50 percent. DVT is a common complication after gastrointestinal tumor surgery, and proper nursing care is essential to lowering the risk of VTE. This research was thus done to examine if intensive nursing interventions may reduce the risk of lower limb DVT in elderly patients who had undergone surgery for gastrointestinal malignancies. The data is separated into two categories: control and treatment. As a self-care theory-based intervention strategy, we propose a hybridized KAP (knowledge, attitude, and practice) approach. Using the twin-bound decision tree algorithm (TBDTA), clinical outcomes including survival and patient satisfaction are examined. There was a considerable improvement in the treatment of DVT compared to the control group and a decrease in typical postoperative conditions. The bundles of care treatment have made a significant increase in the quality of nursing care.

## 1. Introduction

A soft tissue sarcoma that may develop in any part of the digestive system, GISTs (gastrointestinal stromal tumors) can be found everywhere. One of the most common targets is the stomach or small intestines. GISTs originate in the digestive tract's specialized nerve cells, where they spread throughout the body. In the autonomic nervous system, these cells may be found. A change in the DNA of one of these digestive-controlling cells results in the development of a GIST. It is possible for small GISTs to produce no symptoms and to develop at a slow enough pace to have no substantial impact on the body. A fast-bleeding tumor is a common reason for people with big GISTs to seek medical attention when they vomit or urinate blood. GIST cancer is treated mostly by surgery. In the days and weeks after surgery, patients are more likely to develop deep vein thrombosis (DVT). A thrombus or blood clot is formed in a deep vein with this disease. The most common location for them is on the leg. In contrast, a deep vein thrombosis (DVT) may develop in the arm or any other part of the body with a deep vein. A portion of the clot that escapes from the vein and makes its way to the lungs is known as an embolus. Pneumonic embolisms (PEs) occur when blood vessels in the lung get clogged [1].

Deep venous thrombosis (DVT) in the lower extremities is the most prevalent cause of pulmonary thromboembolism (PE), the second leading cause of mortality in cancer patients. There is a common term for both PE and DVT, which are considered sequential diseases, and they are combined to form venous thromboembolism (VTE). A frequent side effect of surgery is deep venous thrombosis (DVT), an intravenous clot-occlusive condition. Lower limbs, particularly the left, are affected. Generally, it may lead to lower-extremity thrombosis and pulmonary embolism, which can even occur in more severe forms of the condition. Patients with malignancies, chronic illnesses, or those who have had significant surgery may be at risk for developing deep vein thrombosis (DVT) [2].

Upper and lower DVT is the development of a thrombus in the deep veins of the upper or lower extremity, depending on location. Deep veins of the upper extremity include the forearm's ulnar, radial, and interosseous veins, as well as the brachial and axillary veins. There are two forms of DVT in the lower limbs: distal vein thrombosis and proximal vein thrombosis. The lower leg and calf are included in the distal part. Proximal veins include the popliteal, femoral, and iliac veins [3].

In any given year, there are 95 new cases per 100,000 people. The most prevalent long-term consequence of DVT is a postthrombotic syndrome (PTS), which is defined as persistent venous symptoms and/or signs as a result of DVT. This occurs in 20 to 50 percent of patients after two years. PTS patients often experience limb discomfort, edoema, and cramping. When standing or walking, these symptoms worsen and improve with rest and supine position. Approximately 2% to 30% of individuals with symptomatic DVT develop severe PTS, which is defined by the development of painful venous ulcers. As a result, PTS has a demonstrable negative influence on mortality and well-being. Seventy-two percent of those who are autopsied had lower levels of DVT. Approximately 50,000 to 200,000 people die each year from pulmonary embolism, the most dangerous result of deep vein thrombosis. It has been estimated that the incidence of deep vein thrombosis (DVT) after most surgical procedures is roughly 50%.

(i) Underdiagnosed and potentially fatal, deep vein thrombosis (DVT) is a medical disorder that may cause both disability and death. Increased risk of DVT is associated with aging and has been steadily increasing in recent years despite several preventative measures. When it comes to younger patients, women are more likely to be impacted than older patients, but this is reversed when it comes to senior patients. Thrombosis and cancer are linked by a well-known dependency. Cancer patients are three times more likely than noncancer patients to have a fatal pulmonary embolism (PE) as a result of deep vein thrombosis (DVT) [4]

(ii) Pulmonary embolism (PE) and deep vein thrombosis (DVT) are both types of venous embolism (VTE) (DVT). VTE risk is increased in those with a history of cancer or other cancer-related conditions. The risk of developing venous thromboembolism (VTE) is four to seven times greater in cancer patients than in the general population. Another important risk factor for VTE, which may be life-threatening, is surgery. In terms of cancer-related deaths, gastric cancer remains the primary cause globally, and the most promising therapy is radical resection. Retrospective studies have looked at VTE after gastrectomy in great detail [5]

Deep venous thrombosis in the lower limbs in elderly patients with gastrointestinal malignancies following surgery is the focus of this research, which examines the effect of intensive nursing care.  Section 2, which includes references and a problem statement, is the rest of this investigation.  Section 3 explains the process.  Section 4 examines and evaluates the methodology's performance. Finally, in Section 5, the study's principal findings are summarised.

## 2. Related Works

Nursing interventions for deep vein thrombosis of the lower legs in elderly patients with gastrointestinal malignancies after surgery are included in this section.

According to the authors in [6, 7], the patients having neurosurgical operations are at risk for deep vein thrombosis (DVT), which may result in venous thromboembolism (VTE). Preventing DVT is a highly monitored quality metric that is often connected to accreditation, hospital ratings, and reimbursement as a major source of avoidable hospital death. Anticoagulant medications are often used in adult therapy to avoid blood clots. Deep vein thrombosis (DVT) is not characterized in children's hospitals, and the risk or effectiveness of therapy is not well understood. DVT may be less prevalent in children than in adults, despite the lack of prospective evidence. DVT risk in children under the age of 12 is typically regarded to be very low.

Deep vein thrombosis (DVT), according to the author in [8] is a common side effect of cancer treatment. There is a significant postoperative rate of DVT after surgery for colorectal cancer (CRC), although the preoperative rate and risk factors have yet to be fully elucidated. The purpose of this retrospective research was to examine the prevalence and risk factors for DVT in patients undergoing CRC surgery in the hospital before the procedure.

There was a study in [9] that sought to determine the effectiveness of screening lower extremities for deep venous thrombosis (DVT) and early care in decreasing cases following major intestinal surgery (MIS) for malignancy of the veins of the stomach.

An investigation on the predictive utility of TEG for lower extremity deep venous thrombosis (LDVT) after surgery in patients with stomach cancer and portal hypertension is presented by the author [10] in this article.

Although upper extremity deep vein thrombosis (UEDVT) is rare, it should not be ignored since it may have deadly effects, according to the authors of [11]. Despite reports indicating the use of central venous catheters (CVCs), malignancy, and surgical invasion have all been linked to an increased incidence of UEDVT, little information is available on the effects of esophagectomy. Research in this research aimed at finding out whether clinical variables, such as CVC placement and thromboprophylaxis approach, is associated with an increased risk of UEDVT in patients who have esophageal cancer surgery.

Permanent atrial fibrillation is connected to an increased risk of embolic effects, as discussed by the authors in [12]. The link between pAF and pulmonary embolism (PE) has not been adequately investigated in elderly people. It is the purpose of this research to determine whether or not individuals with pAF are at a greater risk of developing deep vein thrombosis (DVT) (DVT).

An upper limb deep venous thrombosis caused by CVC is described in [13] as a usual complication of CVC in cancer patients. These individuals' risk factors for CVC-related thrombosis are unknown. Enoxaparin for the prevention of CVC-related thrombosis has been studied in a randomized, double-blind, placebo-controlled trial to identify risk factors for CVC-related thrombosis in patients who were included in the study. Mandatory venography was performed after six weeks of study therapy to look for CVC-related thrombosis. Deep vein thrombosis associated with CVC was shown to be associated with several different baseline patient characteristics. A technique known as multiple logistic regression analysis was used to identify risk variables that were not related to each other.

An instance of pulmonary embolism in a gastric GIST is discussed in [14]. It is presently advised that patients with cancer-related thrombosis get anticoagulation with low molecular weight heparin (LMWH). For an indefinite time or until treatment is discovered, long-term anticoagulation should be taken into consideration.

In [15], the authors describe that although the lower limbs are more often affected by VTE, it may also affect the upper limbs, the splenic and cerebral veins, and the arteries of the abdomen. Cancer patients have an increased incidence of VTE. Because of this, it is necessary to identify risk factors for thrombosis in cancer patients to develop effective prophylaxis. Thrombosis is a common complication in cancer patients, and the researchers wanted to find out how often it occurs and what characteristics are related to it.

PE and deep vein thrombosis (DVT) in patients who have undergone urologic tumor surgery are examined by the author in [16]. Postoperative D-dimer was tested to determine whether it may help predict venous thromboembolism events (VTE) and if there were any other risk variables associated with thromboembolism.

In [17], the authors cite numerous risk factors for VTE, including increasing age, venous stasis, malignant disease, long-term immobility and immobility for an extended period, history of VTE, severe infection, and chronic renal failure. Also, mentioned in [17] are the peripartum period, hormone replacement therapy, the use of oral contraceptives, and ovulation-inducing drugs. Before surgery, women with ovarian cancer had little knowledge on how to handle VTE. Studying ovarian cancer patients, researchers wanted to learn more about the risk factors for VTE and how to treat and prevent it throughout the postoperative period.

According to [18], the meningiomas may be aggravated by venous thromboembolism (VTE) in the postoperative period after surgical excision; however, the exact frequency of this occurrence is unclear. The researchers set out to find out whether meningioma patients who had had postoperative clinical and objective VTE screenings developed VTE themselves.

VTE (venous thromboembolism) is the leading cause of morbidity in patients undergoing neurosurgical procedures, according to [19]. If a preoperative DVT screening protocol is implemented for patients having brain tumor surgery, the authors believe that this high-risk subgroup will be better identified as having DVT so that appropriate treatment can be given to minimize their risk of pulmonary embolism (PE) and improve their overall outcomes and quality of care.

In [20], the authors describe a potentially lethal consequence of surgery as venous thromboembolism (VTE). To reduce one's chance of developing deep vein thrombosis (DVT), one must be aware of the risk factors and take appropriate precautions. Patients undergoing surgery for stomach cancer were the focus of their investigation, which sought to identify risk factors for deep vein thrombosis.

Patients and medical professionals alike are at risk for serious complications after elective surgery for degenerative musculoskeletal diseases, as discussed by the authors in [21]. If you are not careful, you might end up with an infection. Before elective surgery for degenerative musculoskeletal conditions, such as TKA, THA, and spinal surgery, and the researchers wanted to perform a cross-sectional analysis of deep venous thrombosis (DVT) and establish the parameters associated with DVT before surgery.

### 2.1. Problem Statement

For the second consecutive year, cancer patients died from venous thromboembolism as the main cause of mortality. In addition, even when anticoagulant medicine is administered, cancer patients are at greater risk of recurrent VTE and major bleeding difficulties. As the most prevalent symptoms of DVT, pain and lower limb oedema are among the most specific. It is common for deep vein thrombosis to occur when a clot develops in one or more of your leg's deep veins (DVT). Deep vein thrombosis is often accompanied by leg discomfort and edoema. Affected limb swelling, discomfort in the affected leg, red or discolored skin on the leg, and a feeling of warmth in the affected leg are all signs of deep vein thrombosis (DVT). DVT may culminate in a potentially fatal complication known as PE. Toxicology is the term used to describe the condition when a blood clot (thrombus) moves from another part of the body and stops a blood artery in the lung. Symptoms of a PE include shortness of breath, coughing up blood, and experiencing chest discomfort when breathing in or coughing. As a consequence, this research examines the lower limb thrombosis-preventative impact of deep vein thrombosis in older individuals.

## 3. Materials and Methods

Data on patients with gastrointestinal tumors are gathered in this area. Patients suspected of having deep vein thrombosis will be analyzed using the data gathered. Both the control and the therapeutic groups of patients suspected of having deep vein thrombosis are separated. The hybridized KAP-self-care theory-based nursing intervention approach was used in the intervention group. A twin-bound decision tree algorithm (TBDTA) is used to evaluate the effectiveness of the intervention.  Figure 1 depicts the study's overall flow.

- Dataset collection

A database of individuals diagnosed with gastrointestinal stromal tumors (GISTs), leiomyoma, leiomyoblastoma, and leiomyosarcoma from September 2011 to December 2019 was retrieved from Sichuan Provincial People's Hospital, China. A pathologist from the Department of Pathology examined their histology slides. Our research included participants who had been diagnosed with GISTs.

Patients' age, gender, comorbidities, and tumor presentation status were all noted. We could assess how much illness and past therapy the patient had when they initially came to our hospital by looking at their tumor's presentation status. The tumor was classified as primary, metastatic, or locally recurrent, depending on how far it had spread. Hemodynamically, significant blood loss was used to characterize acute gastrointestinal hemorrhage as opposed to transfusion-dependent blood loss. Intermittent melena, guaiac-positive stool, or iron-deficiency anaemia were all considered signs of persistent gastrointestinal hemorrhage. These individuals underwent a variety of diagnostic procedures. Barium investigations, endoscopies, and abdominal ultrasonography all used contrast media to examine the digestive system. GISTs were diagnosed in a total of 47 individuals [22].

### 3.1. Patient Characteristics

GIST was discovered in 47 people from September 2011 to December 2019 (26 males and 21 women). This group's average follow-up duration was 31 months (range 0-99 mo). The average age of the population was 66.6 years old (SD 13.1, range 29 to 87). There was a high incidence of tumors in the stomach, followed by the small intestine, oesophagus, omentum, and colon. An abdominal mass and/or bleeding from the gastrointestinal tract were the most prevalent presenting symptoms in our 28 individuals (60 percent) (10 patients, 21 percent). In 47 patients, 23 patients are in the control group and 24 patients are in the intervention group, respectively.  Table 1 and Figure 2 provide an overview of the patients' demographics.

(B) Suspected deep vein thrombosis (DVT)

Your deep veins, most usually in your lower legs, may get blocked by an abnormal accumulation of fibrin (the fibrous material that holds blood together) that forms a blood clot (thrombus). When deep vein thrombosis (DVT) occurs, it may cause swelling or soreness in the limbs, but it can also develop without showing any symptoms at all. We use the information we have gathered to examine deep vein thrombosis (DVT) patients. One of the tests listed below is used to diagnose DVT.

1. D-dimer blood test

Blood clots create D-dimer, a type of protein. D-dimer levels in the blood are almost always elevated in persons with severe DVT. A normal D-dimer test result can often help rule out PE.

(2) Duplex ultrasound

Sound waves are used to create images of how blood flows through your veins in this noninvasive examination. It is the gold standard for detecting DVT. A professional uses a small hand-held device (transducer) to gently slide a small hand-held device (transducer) across your skin across the body area being investigated for the test. A series of ultrasounds may be performed over several days to assess whether a blood clot is developing or whether a new one has formed.

(3) Venography

In your foot or ankle, a dye is injected into a big vein. To check for clots, an X-ray provides an image of your legs and feet' veins. Because the test is intrusive, it is only used in exceptional circumstances. Other tests, such as ultrasonography, are frequently performed first.

(4) Magnetic resonance imaging (MRI) scan

To identify DVT in the veins of the abdomen, a magnetic resonance imaging (MRI) scan test may be carried out.

Patients who are having less or no symptoms of DVT are in the control group (*n* = 23) and patients with high symptoms of DVT are in the intervention group (*n* = 24).

(C) Control group

The control group is the one in an experiment that is free of intervention by the researchers. The control group patients do not receive any medication that the researchers are studying. Control group patient receives ordinary care.

(D) Intervention group

The intervention group is the one in which the medicine, vaccination, or other intervention being evaluated is administered to the patients. Aside from medical procedures (such as radiation therapy and surgery), medical equipment, behavior modifications (such as diet and exercise), education programs, and counselling are also examples of interventions that may be used. It is referred to as an experimental group or an exploratory group. The patients in the intervention group undergone hybridized KAP-self-care theory-based nursing intervention model.

(E) Hybridized KAP-self-care theory-based nursing intervention model

In the hybridized KAP-self-care nursing paradigm, knowledge (K), attitude (A), and practice (P) are all abbreviated (P). It is the purpose of the hybridized KAP-self-care nursing approach to help patients get a better understanding of their condition so that they may make healthier lifestyle choices in their daily lives. Those in the control group were given the usual nursing services. The intervention group was given the hybridized KAP-self-care nursing model based on conventional nursing practices [4].

Patients undergoing gastrointestinal cancer surgery may expect to receive health education from educators trained in the KAP approach. There was a lot of information about the causes of gastrointestinal cancer, as well as an explanation of the necessity for extreme surgery and the postoperative rehabilitation procedure. By securely embedding gastrointestinal cancer-related knowledge into the brains of patients, it has a modest influence on the emergence of positive behavior for disease rehabilitation. Patients with gastrointestinal cancer who used this approach had considerably better overall health scores than those in the control group throughout the perioperative period, which suggests that it was successful in raising compliance and resulting in more active participation in treatment. It is worth promoting the hybridized KAP-self-care model is widely in clinical use because, in comparison to traditional health education, it emphasizes feedback from information recipients and whether patients understand and can apply knowledge transferred by nurses, as well as the positive effects of health education on patient behavior. Nursing education and experience are critical to the model's success, but so is a professional mindset [5].

To protect the physical and psychological well-being of patients during the perioperative period, the safe management model requires strict adherence to a variety of rules and regulations, as well as operational protocols. Patients' comprehension of self-care and protection of their rights have made the safe nurse management model an essential part of clinical nursing practice. Postoperative rehabilitation training was guided by detailed descriptions of safe rehabilitation exercises, while the quality of nursing care required that the nursing staff standardize and plan their work. Nursing staff safety and service expertise are also promoted by the safe nursing model, which improves patient recovery.

### 3.2. Case Nursing Model

Since its beginnings in social work management, case management has been widely embraced by healthcare professionals in the United States, where it has witnessed enormous growth. Additional qualifications for the post were a case manager with more than eight years of experience, a bachelor's degree, and other relevant abilities. Patient data gathering, nursing plan preparation, stage-based patient monitoring, and guidance, as well as continuous nursing measures (telephone follow-up visits, QQ group organization, and publicizing of the case manager's telephone number), were all part of the case management. During the perioperative phase for gastrointestinal cancer surgery, a one-on-one full-course nursing strategy was used. For the duration of the operation, this method was employed in concert with primary holistic nursing to guarantee that the nursing process remained uninterrupted. Even after patients left the hospital, case managers maintained in touch with them and offered phone consultations for up to six months after they were released. They say that case nursing helps patients with gastrointestinal cancer take advantage of the skills and resources available to them while also reducing any uncertainty they may have had about their condition during treatment, which ultimately leads to better overall patient satisfaction. As a result of their worry of cancer recurrence, patients have been shown to feel more anxious when they are reexamined and follow-up visits are required, according to several studies. For the most part, female cancer survivors discover their relapses, and many are under the mistaken assumption that attending further visits would provide them any additional tools for adjusting to life after cancer treatment. There is a belief among many patients that, although the hospital administers prescription medicines, there is no treatment that can restore their health.

(F) Analysis of the efficiency of intervention by using twin-bound decision tree algorithm (TBDTA)

Both the control and intervention groups are examined in this research using the twin-bound decision tree algorithm. Twin-bound decision tree algorithm is one of the most often used statistical modeling techniques. Data mining and machine learning are further uses for it. It uses a decision tree to make inferences about an object's expected to result from its observations (also known as a predictive model). Classification is a term used to describe the process of dividing up the whole data set used in the procedure. For each component in a given area, many classes are utilized to characterize them. Each inner (nonleaf) hub of an ordered (twin-bound) decision tree is labeled with the information it holds. As a consequence of previous nodes, each node offers information about the anticipated information or the outcome of each instance. Class or probability distribution labels appear on each leaf of this tree, indicating which class or probability distribution each piece of data belongs to. This is how the tree categorizes and organizes the data. It worked by separating the source set, which contained the tree's root hub, into subsets that were then utilized to generate the tree's child nodes. Numerous separation rules are based on arrangement properties and use those traits to define separating.

It is defined as “the complete reduction in the variance of the target variable *y* due to a split at this node,” according to equation (1).

(1) $$\begin{array}{c} I_{V}\left(M\right)=\frac{1}{{\left|s\right|}^{2}}\underset{i\epsilon S}{\sum }\underset{j\epsilon \text{S}}{\sum }\frac{1}{2}{\left(y_{i}-y_{j}\right)}^{2}\left(\frac{1}{\left|\text{st}\right|2}\underset{i\epsilon St}{\sum }\underset{j\epsilon \text{St}}{\sum }\frac{1}{2}{\left(y_{i}-y_{j}\right)}^{2}\right)+1\text{Sf}2i\epsilon S\text{f}J\epsilon \text{Sf}12\left(y_{i}-y_{j}\right)2. \end{array}$$

When a decision tree is constructed, the relevance of each characteristic is determined as shown in equation (2).

(2) $$\begin{array}{c} {fi}_{i}=\frac{\sum_{j:\text{node }j\text{ splits on feature }i}{qi}_{j}}{\sum_{k\in \text{all nodes}}{qi}_{k}}. \end{array}$$

The homogeneity of a sample may be determined using a twin-bound decision tree, which uses entropy to do so. It is 0 if the sample is homogenous, and one if the sample is evenly split. If the sample is not evenly divided, the entropy is one.

In equation (3), entropy is calculated by employing the frequency table of a single attribute:

(3) $$\begin{array}{c} E\left(S\right)=\overset{c}{\underset{i=1}{\sum }}-r_{i}\log_{2}r_{i}. \end{array}$$

The frequency table of two attributes [1] is used to calculate entropy, as illustrated in equation (4).

(4) $$\begin{array}{c} E\left(T,X\right)=\underset{c\in X}{\sum }R\;\left(c\right)E\left(c\right). \end{array}$$

To compute Gini debasement for a lot of things with *J* classes, assume *i* ∈ {1, 2, ⋯.., *J*}. And let *P*_*i*_ be the fraction of items labeled with class *i* in the set as in equation (5).

(5) $$\begin{array}{c} I_{G}\left(R\right)=\overset{J}{\underset{i=1}{\sum }}R_{i}\underset{k\neq i}{\sum }RK=\overset{J}{\underset{i=1}{\sum }}R_{i}\left(1-R_{i}\right)=\overset{J}{\underset{i=1}{\sum }}\left(R_{i}-{R_{i}}^{2}\right)=\overset{J}{\underset{i=1}{\sum }}R_{i}-\overset{J}{\underset{i=1}{\sum }}{R_{i}}^{2}=1-\overset{J}{\underset{i=1}{\sum }}{R_{i}}^{2}. \end{array}$$

This is dependent on the concept of entropy and the data content from the data hypotheses, which are both important. According to equation (6), entropy is defined as follows:

(6) $$\begin{array}{c} H\left(T\right)=I_{E}\left(R_{1}R_{2},\cdots ,R_{J}\right)=-\overset{i}{\underset{i=1}{\sum }}R_{i}\log_{2}R_{i}. \end{array}$$

The fractions *R*_1_, *R*_2_, ⋯, {\*R*_1_, *R*_2_, ⋯} *R*_1_, *R*_2_, ⋯ add up to 1 and represent the proportion of each class present in the child note that results from a split in the tree described in equation (7).

(7) $$\begin{array}{c} IG\left(T,a\right)=H\left(T\right)-H\left(T\;|\;a\right)=-\overset{j}{\underset{i=1}{\sum }}R_{i}\log_{2}R_{i}-\underset{a}{\sum }R\left(a\right)\log_{2}Rk\left(i\;|\;a\right). \end{array}$$

As shown in method 1 (Algorithm 1) below, the technique for constructing a twin-bound decision tree is straightforward.

## 4. Result and Discussion

In this phase, we are going to explain the clinical analysis of vein thrombosis by employing the twin-bound decision tree approach. The findings of the proposed approach are depicted by utilizing the MATLAB tool.

The total incidence of symptomatic DVT was substantially lower in the intervention group (2.2 percent) than in the control group (7.4 percent); however, there was no significant difference in the incidence of symptomatic PE between the two groups (1.5 percent vs. 3.7 percent) in Figure 3. There was no significant difference in the site of DVT between the two groups. No life-threatening PE or death developed in the trial group. Meanwhile, of the four patients with life-threatening PE in the control group (0.9 percent), two subsequently expired due to significant progression (0.5 percent).

Figure 4 depicts the distribution of lower deep vein thrombosis. CPV denotes the common femoral vein, DFV denotes the deep femoral vein, PV denotes the peroneal vein, ATV denotes the anterior tibial vein, and PTV denotes the posterior tibial vein. Lower extremity deep vein thrombosis affects these veins.

Figure 5 demonstrates that respondents had a generally good view of VTE treatment: almost 70% said the treatment was beneficial and safe, and they were in favor of obtaining it. However, just around half of those who received the medication said the side effects were manageable. The majority of responders (78%) were happy with the treatment time; however, only 56 and 46 percent were happy with the information they received concerning the treatment and DVT/PE, respectively. In Figure 5, A indicates that the injection timing was acceptable, B indicates that the rationale for the injection was sufficiently stated, and C indicates that the information provided on DVT/PE was satisfactory.

Figure 6 depicts the risk of VTE in cancers of the pancreas, lungs, GI tract, liver, bladder, kidney, and uterine.

Figure 7 shows that during the first six months of follow-up, the risk for both cohorts was three times the predicted level, after which it fell to a consistent level of slightly more than 1.0 one year after the thrombotic event and throughout the research period.

## 5. Conclusion

Patients who have had gastrointestinal tumor surgery are the focus of this investigation. The most common form of therapy for an intestinal tumor is surgery. In the days and weeks after surgery, patients are at significant risk of developing a deep vein thrombosis (DVT). Patients with tumors or those having major surgery have an increased risk of developing deep vein thrombosis, which may be life-threatening. Your deep veins, most usually in your lower legs, may get blocked by an abnormal accumulation of fibrin (the fibrous material that holds blood together) that forms a blood clot (thrombus). A focus on providing care that is personalized for each patient is a cornerstone of the nursing profession. Patients with gastrointestinal cancers have been the subject of several studies on the use of quick rehabilitative nursing. Rapid postoperative recovery of intestinal function, increased nutrition, lessened negative emotions, enhanced quality of life, and fewer complications are all benefits of accelerated rehabilitation nursing care for gastrointestinal tumors. As a result, we propose a hybridized KAP (knowledge, attitude, and practice) self-care theory-based intervention approach for the treatment group in our research. Utilizing the twin-bound decision tree algorithm (TBDTA), clinical outcomes including patient survival and satisfaction are evaluated.

## Figures and Tables

**Figure 1:** Flow of the suggested methodology.

**Figure 2:** GIST location.

**Figure 3:** Incidence of venous thromboembolism events and mortality.

**Figure 4:** Distribution of lower extremity deep veins.

**Figure 5:** VTE satisfaction.

**Figure 6:** Absolute rate of venous thromboembolism (VTE) by various cancer.

**Figure 7:** Risk of DVT or PE.

**Algorithm 1:** Twin-bound decision tree algorithm (TBDTA).

**Table 1:** Characteristics of a patient.

Characteristics	*n* (%)
Number of patients	47
Male/female (ratio)	26 : 21 (1.23 : 1)
Mean age at the time of diagnosis(SD)	66.60 (SD 19.1)
Median follow-up time in months(IQR)	26.00 (10-43)
Presenting symptoms GI bleeding Epigastric pain Abdominal mass Incidental finding	28 (60%) 21 (45%) 10 (21%) 3 (6.3%)
Locations Stomach Small bowel Esophagus Colon Omentum	34 (72.3%) 8 (17.0%) 2 (4.3%) 1 (2.1%) 2 (4.3%)
Death Total Tumor related Tumor unrelated	16 (34%) 11 (23.4%) 5 (10.6%)

## Data Availability

The analyzed datasets generated during the study are available from the corresponding author on reasonable request.
